The article "Situation Element Extraction Based on Fuzzy Rough Set and Combination Classifier" was published in 2022. Journal: Comput Intell Neurosci.

# Situation Element Extraction Based on Fuzzy Rough Set and Combination Classifier

**DOI:** 10.1155/2022/3429227

**Published:** 2022-08-23

**Authors:** Dongmei Zhao, Hongbin Wang, Yaxing Wu

**Affiliations:** ^1^College of Computer and Cyber Security, Hebei Normal University, Shijiazhuang, China; ^2^, Hebei Key Laboratory of Network and Information Security, Shijiazhuang, China; ^3^Hebei Provincial Engineering Research Center for Supply Chain Big Data Analytics & Data Security, Shijiazhuang, China

## Abstract

Generalized network security situation awareness technology is divided into three processes: situation element extraction, situation understanding, and situation prediction. Situation element extraction is the most critical step in the whole process, and its extraction quality will directly affect the accuracy of situation understanding and prediction. In view of the shortcomings of current situation element extraction methods, this study makes an in-depth study on the network security situation element extraction algorithm and proposes a situation element extraction model based on the fuzzy rough set and combined classifier, which is used to improve the accuracy of situation elements acquisition, so as to provide a better data basis for situation understanding and prediction. In this study, the theory of fuzzy rough set is used to reduce the attributes of data without reducing the ability of data classification, which reduces the complexity of data; using the combination classifier theory and particle swarm optimization algorithm, a framework of situation element extraction is built, which can extract situation elements more accurately. The experimental results show that the network security situation element extraction framework proposed in this study can effectively shorten the extraction time of situation elements and improve the accuracy of situation element acquisition under the premise of ensuring the ability of data classification, thus proving the effectiveness and feasibility of the situation element extraction framework proposed in this study.

## 1. Introduction

With the gradual expansion of the scope of the network, the amount of information generated on it is increasing. With the development of network, the security threats caused by the network are increasing and more complex. The network attacks against these security problems are also increasing and more complex. As a result, the network intrusion detection and defense system based on passive defense and other network security devices are tired of coping with such a large number of complex network attacks. Even though there are many passive security products on the network, they are like isolated islands, fighting on their own, and lacking necessary communication and cooperation [1] and cannot play a very good effect on complex, multi-step, and hidden attacks. Network security situation awareness technology can quickly and accurately identify the type of attack and predict the attack intention, so that network managers can respond in time to avoid greater losses. Because of the great advantages of network security situation awareness technology, it has been the focus of the majority of scholars since its birth. The extraction of network security situation elements is the basis of the perception process, and the accuracy of the whole perception process will be directly affected by its extraction accuracy.

Network security situational elements refer to elements or attributes that can reflect the current security state of the network; that is, the current network state can be inferred through the changes in these elements or attribute values, and situational element extraction is to use extraction technology to extract these situational elements from the multisource heterogeneous network security information generated by a large number of network security devices which is accurately extracted. The first step in network security situational awareness is to extract situational elements, and the quality of the extracted elements will directly affect the accuracy of situational understanding and prediction. Situational elements are extracted from information sources, and the extracted situational elements must meet the requirements of being accurate, comprehensive, easy to extract, and highly recognizable. According to the different sources of security data information, we can divide the network situation elements into three parts: basic network environment elements, security vulnerability elements, and attack information elements. Basic network environment elements refer to the elements that reflect the configuration of the network and various network access devices, network topology, etc.; security vulnerability elements refer to the elements that reflect the vulnerability of the network, that is, information that can reflect the inherent defects of the network or equipment. Element: attack information element refers to the element that reflects the type of attack the network is currently receiving. It can be seen from the above explanation that the basic network environment elements and security vulnerability elements are inherent information of the network itself. They can only reflect the hidden dangers existing in the current network and possible attacks and cannot directly affect the change in network security status. Information elements can not only directly reflect the current network security situation but also reflect the network loopholes and hidden dangers. Therefore, the extraction of attack information elements is the most important part of network situation element extraction. In the face of increasing network data, it is of far-reaching significance to study how to remove redundant information from it and extract comprehensive and accurate situation elements [2].

In the aspect of network security situation awareness, Endsley first put forward the concept of situation awareness in 1988 and established a three-layer awareness model [3]. In 1999, Bass introduced it into the field of network security and then established a JDL model based on data fusion [4]. Since then, the active network defense technology has developed rapidly in the field. Liu and others combined evidence theory with particle swarm optimization to build a hierarchical situation awareness model [5]. Leau et al. constructed a hierarchical evaluation mechanism based on entropy and a network situation awareness mechanism based on the Grey Verhulst–Kalman prediction [6]. Zhang et al. introduced the stochastic game theory into situation awareness and quantified the situation value through the game effectiveness of both sides in the cloud computing environment [7]. Chen et al. constructed a network situation awareness model using a variable step learning mechanism and simulated annealing method to optimize BP neural network [8]. Liu et al. used different weights to fuse data sources, quantified situation value with the hierarchical method, and realized automatic control of network security situation awareness by applying cognitive awareness for the first time [9]. Li and Duan optimized the hidden Markov model with the crowd search method and realized effective situation evaluation [10]. He and Zhu combined the GRU neural network and particle swarm optimization method to mine the time relationship of data, used the attention mechanism to measure the situation value of current network, and constructed a neural network situation awareness model with the attention mechanism [11]. Samuel effectively combines a decision tree and artificial neural network to build an enhanced network situation awareness model [12]. The authors have also done some in-depth research in the field of network security situational awareness and achieved a series of relevant results [13–17].

In the aspect of fuzzy rough set theory, in 1990, Dubois and Prade first proposed the concepts of rough fuzzy set and fuzzy rough set [18] and published a monograph on fuzzy rough set in 1992 [19]. Since then, fuzzy rough set theory has become the main attribute reduction method. In 2011, Chen et al. introduced the Gaussian kernel function into fuzzy rough set theory, described the similarity of fuzzy attributes with the Gaussian kernel, and constructed an attribute selection algorithm based on the difference matrix [20]. In 2019, Wang et al. added a distance measurement index in fuzzy rough set theory and used variable distance to measure the importance of attributes, so that the attribute reduction was completed with the variable distance measure function [21]. Senthilnayaki et al. introduced the maximum correlation algorithm to fuzzy rough set theory for attribute reduction and then used the improved k-nearest neighbor algorithm to extract situation elements [22], which effectively reduced the false alarm rate of attacks. In 2020, Ghoutkhar and Nehi have effectively integrated the traditional rough set theory and the regional value fuzzy set theory and put forward a general method of selecting fuzzy rough set attributes and a new development direction [23]. In the same year, Ni and others designed a dynamic attribute reduction algorithm, which added an incremental mechanism on the basis of fuzzy rough set theory, which can dynamically and quickly update the attributes based on the existing attribute selection results [24].

In terms of combined classifiers, Hansen's and Salamon's paper published in 1990 shows that different classifiers can provide complementary information for sample classification [25]; that is to say, using multiple classifiers for fusion classification can improve the performance of classification system, which lays a foundation for the development of combined classifiers. In 1998, Kittler and others deeply studied the combined classifier, gave the specific framework of the model for fusion classification, and defined two fusion methods based on the sum rule and product rule [26]. Since then, the theory of combined classifier has gradually developed and become a research hotspot in various fields. In 2002, Ma carried out in-depth research on combined classifiers and proposed two classifier set selection methods based on minimum dependency and genetic algorithm [27]. Then, the results of classifier set generation were fused with a neural network to improve the accuracy of system classification. In 2003, Giacinto and others constructed a combined classifier fusion model to detect network intrusion [28]. In 2008, Wang and others proposed the hierarchical model of situation awareness and applied the combination classifier fusion method [29] at each level, which achieved good results in situation understanding and prediction. In 2016, Mi et al. applied the weighted vector to the fusion layer of the combined classifier and then used the k-nearest neighbor algorithm to adjust the misclassified samples [30], thus improving the classification performance. In 2019, Mo and Ma constructed a new value integral algorithm [31] based on the value integral algorithm of fuzzy sets and applied the algorithm to the fusion layer of combined classifiers, which greatly improved the recognition ability of combined classifiers. In 2020, TTN and others used the interval to represent each category of data, trained the combined classifier, and then used PSO algorithm to find the optimal parameters of fusion [32], which improved the accuracy of fusion recognition. In 2021, Wang et al. constructed a regularized combined classifier based on the random gradient descent algorithm and then determined the fusion weight [33] using the geometric structure of the data set to prevent the overfitting of the combined classifier.

The author analyzes and summarizes the shortcomings of existing research methods. Aiming at some problems faced in the process of situation element extraction, this study focuses on the fuzzy rough set theory and combined classifier theory. In the process of attribute reduction, the fuzzy rough set theory is introduced and effectively improved, and some new measurement indexes and methods are added, and the reduced attributes are made more in line with the actual situation; in the process of extracting situation elements, the combined classifier theory is introduced to make up for the low accuracy of extracting elements by a single classifier. Finally, the improved compression factor particle swarm optimization method based on random vector is used to train the BP network as the fusion layer to make the extracted situation elements more accurate and provide a good data basis for situation understanding and prediction and improve the accuracy of situation understanding and prediction. It can be seen from the results that the situation element extraction framework designed in this study not only improves the accuracy of situation element acquisition but also reduces the operation time, which verifies the advantages of this framework.

## 2. Design of Attribute Reduction Method

If you want to use the classical rough set to deal with continuous data, you must discretize it, but some original data information will be lost. The traditional fuzzy rough set can overcome the above problems, but it only reduces attributes according to the dependence of decision attributes on conditional attributes and does not consider the redundancy of conditional attributes, the maximum membership of samples belonging to real categories, and the influence of noise samples on classification results. Aiming at the shortcomings of traditional fuzzy rough sets, this study proposes a method of attribute secondary reduction based on conditional attribute similarity and maximum similarity criterion, which can delete redundant conditional attributes while ensuring the breadth of classification information. To reduce the influence of noise samples and ensure that the samples belong to the real category of membership, this study proposes an approximate calculation method based on k-order weighted average in the nearest neighbor region, which makes the attribute reduction more accurate and improves the accuracy of situation element extraction.

### 2.1. Attribute Secondary Reduction Method

To reduce the similarity between the condition attributes in the attribute subset after reduction and ensure the information breadth of the subset, a similarity measure method of condition attributes and an attribute selection method based on the maximum similarity criterion are proposed to delete redundant condition features, so as to achieve the goal of attribute secondary reduction.

#### 2.1.1. Similarity of Conditional Attributes

For the similarity measurement between samples and the contribution of conditional attributes to decision attributes, experts and scholars have proposed some classical measurement methods, but there is no unified measurement method for similarity of conditional attributes. This study draws on the experience of similarity between samples and the contribution of conditional attributes to decision attributes, and the similarity measurement methods between discrete and continuous attributes are proposed.

For discrete attributes, we can measure the importance of conditional attributes to decision-making attributes by contributing to classification, which is defined as follows.

**Definition 1 .**

Let the decision system be *S* = *S*={*U*, *C*, *D*, *V*, *f*}, and given the discrete characteristic *cεC*, then the importance of characteristic *c* to *D* can be expressed as follows:

(1) $$\begin{array}{c} s\left(c,D\right)=\frac{\left|\left\{c\right\}\cup D\right|}{\sqrt{\left|\left\{c\right\}\right|}\cdot \sqrt{\left|D\right|}}, \end{array}$$

where |·| is the square sum of the number of objects in each class divided by feature set , that is, the classification degree of features.

Based on the above idea, we can define the similarity between discrete conditional features by different classification degrees of discrete conditional features.

**Definition 2 .**

Let *S*={*U*, *C*, *D*, *V*, *f*} be the decision system and *C*={*c*_1_, *c*_2_, *c*_3_,…, *c*_*m*_} be the conditional feature set. Given discrete features *c*_*k*_, *c*_*l*_ ∈ *C*(1 ≤ *k*, *l* ≤ *m*), the similarity of features c_k_ and c_l_ can be measured by the following formula:

(2) $$\begin{array}{c} s\left(c_{k},c_{l}\right)=\frac{\left|\left\{c_{k}\right\}\cup \left\{c_{l}\right\}\right|}{\sqrt{\left|\left\{c_{k}\right\}\right|}\cdot \sqrt{\left|\left\{c_{l}\right\}\right|}}. \end{array}$$

According to formula (2), if the classification degree of features *c*_*k*_ and *c*_*l*_ is the same, then $\left|\left\{c_{k}\right\}\cup \left\{c_{l}\right\}\right|=\sqrt{\left|\left\{c_{k}\right\}\right|}\cdot \sqrt{\left|\left\{c_{l}\right\}\right|}$; that is, similarity *s*(*c*_*k*_, *c*_*l*_)=1; if the classification degree of features *c*_*k*_ and *c*_*l*_ is different, then $\left|\left\{c_{k}\right\}\cup \left\{c_{l}\right\}\right|<\sqrt{\left|\left\{c_{k}\right\}\right|}\cdot \sqrt{\left|\left\{c_{l}\right\}\right|}$; that is, similarity *s*(*c*_*k*_, *c*_*l*_) < 1.

Assuming that there are only two discrete conditional features of *c*_1_ and *c*_2_ in four samples, the optimal situation is that *c*_1_ and *c*_2_ cannot effectively classify the samples, but the combination can completely classify the samples. The four samples are (0,0), (0,1), (1,0), and (1,1); then, $s\left(c_{1},c_{2}\right)=1^{2}+1^{2}+1^{2}+1^{2}/\sqrt{2^{2}+2^{2}}\cdot \sqrt{2^{2}+2^{2}}=0.5$, and the similarity of the two features is the minimum.

When the conditional features are continuous features, the similarity between features cannot be measured by the classification degree of features. Because if we do not discretize the continuous features, we cannot describe the classification degree of the features by the values of the continuous features. This study uses the experience of distance-based similarity measurement between samples for reference and finds that the similarity between continuous features can be effectively measured according to the distribution of eigenvalues, so a method of measuring the similarity between continuous features according to the distribution of features is proposed.

**Definition 3 .**

Let *S*={*U*, *C*, *D*, *V*, *f*} be the decision system, *U*={*x*_1_, *x*_2_, *x*_3_,…, *x*_*n*_} be the sample set, and *C*={*c*_1_, *c*_2_, *c*_3_,…, *c*_*m*_} be the conditional feature set, and given continuous features *c*_*k*_, *c*_*l*_ ∈ *C*(1 ≤ *k*, *l* ≤ *m*), then the similarity between features c_k_ and c_l_ can be expressed as follows:

(3) $$\begin{array}{c} s\left(c_{k},c_{l}\right)=\frac{\sum_{i=1}^{n}\left|x_{ik}-{\bar{a}}_{k}\right|\cdot \left|x_{il}-{\bar{a}}_{l}\right|}{\sqrt{\sum_{i=1}^{n}{\left(x_{ik}-{\bar{a}}_{k}\right)}^{2}}\cdot \sqrt{\sum_{i=1}^{n}{\left(x_{il}-{\bar{a}}_{l}\right)}^{2}}}, \end{array}$$

where *x*_*ik*_ is the value of the *k*th feature of the *i*th sample in the sample set *U*, and ${\bar{a}}_{k}$ is the average value of the *k*th feature in the conditional feature set; that is, ${\bar{a}}_{k}=1/n\sum_{i=1}^{n}x_{ik}$.

According to formula (3), if the value distribution of the two features is the same, then $\sum_{i=1}^{n}\left|x_{ik}-{\bar{a}}_{k}\right|\cdot \left|x_{il}-{\bar{a}}_{l}\right|=\sqrt{\sum_{i=1}^{n}{\left(x_{ik}-{\bar{a}}_{k}\right)}^{2}}\cdot \sqrt{\sum_{i=1}^{n}{\left(x_{il}-{\bar{a}}_{l}\right)}^{2}}$; that is, the similarity of the two features is *s*(*c*_*k*_, *c*_*l*_)=1; if the distribution is different, the similarity of the two features is *s*(*c*_*k*_, *c*_*l*_) < 1.

#### 2.1.2. Attribute Cyclic Secondary Reduction Based on Maximum Similarity Criterion

After the matrix of attribute similarity is calculated according to the formula of conditional attribute similarity, we can see the correlation between attributes.

To reduce the secondary conditional attributes under the condition of ensuring the information breadth, we first cluster the attributes with high similarity by the direct clustering method and then select representative conditional attributes according to the maximum similarity criterion, so as to realize the secondary reduction of conditional attributes. Finally, the advantages and disadvantages of the secondary reduction attribute set are measured according to the attribute dependency index. Thus, it is decided whether the attribute reduction is needed again.  Figure 1 shows the specific process of conditional attribute reduction.

1. Conditional attribute clustering using the direct clustering method:  the calculation process of direct clustering method is simple and easy to implement, which can save the clustering time of conditional attributes. Therefore, this study uses this method to cluster similar conditional attributes. The specific process is introduced as follows:

**Definition 4 .**

In universe *U*, a sequence of weighted values composed of a group of elements can be called a path:

(4) $$\begin{array}{c} R_{i}=x_{i1}\overset{c_{i1}c_{i2}}{⟶}x_{i2}\cdots x_{i\left(t-1\right)}\overset{c_{i\left(t-1\right)}c_{it}}{⟶}x_{it}, \end{array}$$

  where *R*_*i*_(*i*=1,2,3,…) is the *i*th path in the object set, *x*_*ik*_(*k*=1,2,3,…, *t*) is the *k*th element in the *i*th path, and *x*_*i*1_ and *x*_*it*_ are the starting point and ending point of the *i*th path, respectively. If two roads have the same starting point and ending point, they are considered to be equivalent. An element can appear many times in the path, but it cannot make the path form a loop. Each arrow in the path represents a step in the path, and *c*_*i*(*k* − 1)_*c*_*ik*_(*k*=1,2,3,…, *t*) on the arrow represents the cost or weight of each step.

**Definition 5 .**

The weight of the path is equal to the minimum weight of the step in the path:

(5) $$\begin{array}{c} W_{R_{i}}=\min\left(c_{i1}c_{i2},c_{i2}c_{i3},\ldots ,c_{i\left(t-1\right)}c_{it}\right). \end{array}$$

**Definition 6 .**

The decision system is *S* = {*U*, *C*, *D*, *V*, *f*}, *C* = {*c*_1_, *c*_2_, *c*_3_,…, *c*_*m*_} is the conditional feature set, and *c*_*k*_, *c*_*l*_ ∈ *C*(1 ≤ *k*, *l* ≤ *m*) are given. If there is a path in the conditional feature similarity matrix with *c*_*k*_ as the starting point (or endpoint) and the weight of *c*_*l*_ endpoint (or start point) is not less than *λ*, then *c*_*k*_ and *c*_*l*_ belong to the same class under threshold *λ*. According to the weight definition of the path, the weight of all steps in the path is not less than *λ*, so all elements in the path belong to the same class under the threshold of *λ*.

  According to Definition 6, the conditional feature set can be divided into several feature equivalence classes. However, the same feature attribute may belong to different feature equivalence classes at the same time. For those feature equivalence classes whose intersection is not an empty set, they should be combined into one class to get the final feature equivalence class.
(2) Secondary reduction in conditional attributes based on a maximum similarity criterion
  After clustering the condition attributes with high similarity, a representative condition attribute is selected from the attribute set of each cluster, and other condition attributes are deleted, to achieve a fast reduction in secondary redundant condition attributes. To complete this process, this study proposes a clustering conditional attribute reduction method based on maximum similarity criterion.

**Definition 7 .**

*S*={*U*, *C*, *D*, *V*, *f*} is set as the decision system, *C* is set as the set of conditional attributes, and the similarity matrix of conditional attributes determined by the similarity measurement formula of conditional attributes is SM. Then, according to SM and threshold *λ*, the clustering result of conditional attributes is *C*(*SM*, *λ*)={*C*_1_, *C*_2_, *C*_3_,…, *C*_*r*_} by the direct clustering method, where *C*_*i*_={*c*_*i*1_, *c*_*i*2_, *c*_*i*3_,…, *c*_*is*_}(1 ≤ *i* ≤ *r*) describes the conditional attributes contained in a certain category after attribute clustering, Then, the representative attributes of each clustered category can be expressed as follows:

(6) $$\begin{array}{c} REP_{C_{i}}\left(c\right)=\left\{c_{ik}\in C_{i}|k=\arg\max\left(\left\{vm_{1},vm_{2},vm_{3},\ldots ,vm_{s}\right\}\right)\right\}. \end{array}$$

Among them, argmax({*vm*_1_, *vm*_2_, *vm*_3_,…, *vm*_*s*_}) is the condition attribute index corresponding to the maximum similarity sum of attributes in the set, and *vm*_*j*_ is the similarity sum of the *j*th condition attribute and other condition attributes in the *i*th attribute cluster *C*_*i*_:

(7) $$\begin{array}{c} vm_{j}=\sum_{n=1,n\neq j}^{s}SM\left(c_{j},c_{n}\right),j=1,2,3,\ldots ,s. \end{array}$$

If there are two or more conditional attributes in *C*_*i*_to maximize the total similarity of attributes, then the corresponding conditional attribute with the minimum standard deviation of attribute similarity as the representative attribute is selected, to ensure that the selected conditional attributes represent the corresponding clustering subset of similar attributes to the maximum extent, to reduce the information loss caused by eliminating redundant attributes.

The analysis shows that the number of similar conditional attribute subsets after clustering does not decrease with respect to the clustering threshold, because the reduction process is to select a representative attribute from each similar conditional attribute subset, so the number of conditional attributes in the reduced representative attribute set does not decrease with respect to the clustering threshold; and the more attributes in the reduced representative attribute set, the more decision-making characteristics depend on it [34]. Taking advantage of this phenomenon, we can build a conditional attribute based on the related knowledge in the next section.

### 2.2. Attribute Final Reduction Method

After the redundant conditional attributes are deleted to get the secondary reduction in the conditional attributes, we need to consider the contribution of the conditional attributes to the decision attributes. Some experts and scholars have conducted in-depth research on the importance of conditional attributes to decision attributes as a measure to reduce redundant conditional attributes and put forward some feasible methods. These methods are superior in some aspects, but there are also some shortcomings. In view of the shortcomings of some methods at present, this study redefines the upper and lower approximations of fuzzy rough set theory and proposes a feature selection method of fuzzy rough set based on k-order weighted average.

In Section 2, we have introduced the standard definition of upper and lower approximation of fuzzy rough sets. To facilitate calculation, some experts have given another equivalent definition.

**Definition 8 .**

Let the decision system be *S*={*U*, *C*, *D*, *V*, *f*} and *U* be divided into *r* distinct indiscernible relations {*X*_1_, *X*_2_, *X*_3_,…, *X*_*r*_} by *D*. Given the feature subset *B*⊆*C*, *R*_*B*_ is a binary similar fuzzy relation on the object set *U* under the condition of *B*, and then, the lower and upper approximation sets of *X*_*i*_(1 ≤ *i* ≤ *r*) with respect to *B* are, respectively, expressed as follows:

(8) $$\begin{array}{c} \underline{B}X_{i}\left(x\right)=\underset{y\in X_{i}}{\min}\left\{1-R_{B}\left(x,y\right)|x\in U\right\}, \end{array}$$

(9) $$\begin{array}{c} \bar{B}X_{i}\left(x\right)=\underset{y\in X_{i}}{\max}\left\{R_{B}\left(x,y\right)|x\in U\right\}, \end{array}$$

where $\underline{B}X_{i}\left(x\right)$ is the minimum value of the inconsistency degree of sample *x* ∈ *U* relative to all samples *y* that do not belong to category *X*_*i*_. In other words, $\underline{B}X_{i}\left(x\right)$ depends on the sample *y* that is most similar to x among all samples that do not belong to category *X*_*i*_. $\bar{B}X_{i}\left(x\right)$ is the maximum value of consistency between sample *x* ∈ *U* and all samples *y* belonging to category *X*_*i*_. The above definition uses the fuzzy neighborhood of the sample *x* to measure the importance of the sample to the decision category *X*_*i*_, which is similar to the classical rough set in thought.

Although the above definition can simplify the upper and lower approximation process of fuzzy rough sets and reduce the computational complexity, it does not consider the influence of noise samples on the upper and lower approximation process. If the noise sample *y* is exactly the sample of all samples not belonging to category *X*_*i*_ and the most similar to *x* in the approximate extraction process under category *X*_*i*_, then the lower approximation of *X*_*i*_ obtained at this time is not accurate.

For example, there are two categories of samples in a data set, and the sample distribution is shown in Figure 2. It can be seen that the sample *y*_1_ is far away from its category 2. In this case, it can be considered as a noise sample. When formula (8) is used to calculate the degree that sample *x* belongs to category 1, noise sample *y*_1_ will still be used for calculation, which will lead to an inaccurate calculation of the lower approximation of category 1. However, if *y*_2_ is used to calculate the lower approximation of category 1, more accurate results will be obtained.

To solve the above problems, this study proposes an upper and lower approximation method based on *k*-order weighted average, which can effectively resist the influence of noise samples.

**Definition 9 .**

Let the decision system be *S*={*U*, *C*, *D*, *V*, *f*} and *U* be divided into *r* distinct indiscernible relations {*X*_1_, *X*_2_, *X*_3_,…, *X*_*r*_} by *D*. Given the feature subset *B*⊆*C*, *R*_*B*_ is a binary similar fuzzy relation on the object set *U* under the condition of *B*, and then, the lower and upper approximation sets of *X*_*i*_(1 ≤ *i* ≤ *r*) with respect to *B* are, respectively, expressed as follows.

Let *y*_1_, *y*_2_, *y*_3_,…, *y*_*k*_ be *k* samples with the least degree of inconsistency with sample *x* that are not classified as class *X*_*i*_; then, the lower approximate set of *X*_*i*_(1 ≤ *i* ≤ *r*) about *B* is expressed as follows:

(10) $$\begin{array}{c} \underline{B}X_{i}^{k}\left(x\right)=\left\{\begin{array}{cc} \frac{\sum_{j=1}^{k}{\left(1-R_{B}\left(x,y_{j}\right)\right)}^{2}}{\sum_{j=1}^{k}1-R_{B}\left(x,y_{j}\right)}, & \sum_{j=1}^{k}1-R_{B}\left(x,y_{j}\right)\neq 0,\\ 0, & \sum_{j=1}^{k}1-R_{B}\left(x,y_{j}\right)=0, \end{array}\right\},x\in U. \end{array}$$

Let *z*_1_, *z*_2_, *z*_3_,…, *z*_*k*_ be the *k* samples, which belong to class *X*_*i*_ and are most consistent with sample *x*, and then, the upper approximation set of *X*_*i*_(1 ≤ *i* ≤ *r*) with respect to *B* is expressed as follows:

(11) $$\begin{array}{c} \bar{B}X_{i}^{k}\left(x\right)=\left\{\begin{array}{cc} \frac{\sum_{j=1}^{k}R_{B}{\left(x,z_{j}\right)}^{2}}{\sum_{j=1}^{k}R_{B}\left(x,z_{j}\right)}, & \sum_{j=1}^{k}R_{B}\left(x,z_{j}\right)\neq 0,\\ 0, & \sum_{j=1}^{k}R_{B}\left(x,z_{j}\right)=0, \end{array}\right\},x\in U. \end{array}$$

Firstly, *k* samples that meet the requirements are selected, then the dissimilarity (or similarity) of each sample is multiplied by the corresponding dissimilarity (or similarity) weight, and finally they are added as the final value. By using this method to calculate the upper and lower approximations of fuzzy rough sets, the idea of weighted average can be effectively used to resist the interference of noise. If the sample distribution of a certain data set is shown in Figure 2, the sample *y*_1_ is the noise sample of category 2, and this sample happens to be the sample with the least similarity to sample *x* when calculating the lower approximation of category 1, then this sample must be the sample most similar to category 1 relative to other samples of category 2, that is, relative to other samples of category 2. The similarity weight of the noise sample *y*_1_ is the smallest, so the influence of the noise sample *y*_1_ can be resisted when *k* qualified samples are selected and the lower approximation of category 1 is calculated by the weighted average method.

The approximate decision table under the fuzzy rough set obtained by formula (8) can correctly classify all samples in the example, but it needs to calculate the fuzzy neighborhood of 3^3^=9 samples in the process of obtaining the approximation. If the number of samples in the data set is very large, the calculation time will increase explosively. To effectively reduce the time of calculating the upper and lower approximation of fuzzy rough sets and reduce the influence of noise samples, this study improves the *k*-order weighted average method and proposes a method of calculating the upper and lower approximation of close neighborhood based on order weighted average.

**Definition 10 .**

Let the decision system be *S*={*U*, *C*, *D*, *V*, *f*} and *U* be divided into *r* distinct indiscernible relations {*X*_1_, *X*_2_, *X*_3_,…, *X*_*r*_} by *D*. Given the feature subset *B*⊆*C*, *R*_*B*_ is a binary similar fuzzy relation on the object set *U* under the condition of *B*, and then, the lower and upper approximation sets of *X*_*i*_(1 ≤ *i* ≤ *r*) with respect to *B* are, respectively, expressed as follows:

(12) $$\begin{array}{c} \underline{B}X_{i}^{k}\left(x\right)=\left\{\begin{array}{cc} \frac{\sum_{j=1}^{k}{\left(1-R_{B}\left(x,y_{j}\right)\right)}^{2}}{\sum_{j=1}^{k}\left(1-R_{B}\left(x,y_{j}\right)\right)}, & \sum_{j=1}^{k}1-R_{B}\left(x,y_{j}\right)\neq 0x\in X_{i},\\ 0, & other, \end{array}\right\},x\in U,\\ \bar{B}X_{i}^{k}\left(x\right)=\left\{\begin{array}{cc} \frac{\sum_{j=1}^{k}{\left(1-R_{B}\left(x,y_{j}\right)\right)}^{2}}{\sum_{j=1}^{k}\left(1-R_{B}\left(x,y_{j}\right)\right)}, & \sum_{j=1}^{k}1-R_{B}\left(x,y_{j}\right)\neq 0x\in X_{i},\\ 0, & other, \end{array}\right\},x\in U. \end{array}$$

Among them, *y*_*j*_(1 ≤ *j* ≤ *k*) represents the *j*th sample among the *k* samples that do not belong to category *X*_*i*_ and are least inconsistent with sample *x*, and *z*_*j*_(1 ≤ *j* ≤ *k*) represents the *j*th sample among the *k* samples that belong to category *X*_*i*_ and are most consistent with sample *x*.

Using the above formula to calculate the upper and lower approximations of fuzzy rough sets can ensure that the membership of samples in the category they do not belong to is zero, thus indirectly ensuring that the membership of samples in the real category is the largest. In this way, the method of directly constructing the upper and lower approximations can save most of the unnecessary calculation of the sample fuzzy neighborhood and greatly improve the speed of the upper and lower approximations of fuzzy rough sets. For example, the lower approximation decision table of the data set shown in Table 1 can be obtained using the upper and lower approximation calculation method of the nearest neighbor based on the *k*-order weighted average, which can not only make all samples correctly classified but also only calculate the fuzzy neighborhood of three samples, greatly reducing the calculation time.

Applying the upper and lower approximation calculation method based on *k*-order weighted average to the attribute reduction process of fuzzy rough sets, a heuristic attribute selection algorithm based on addition can be designed for the secondary reduction set of conditional attributes obtained in the previous section. The specific process is shown in Figure 3. Firstly, we take the secondary reduction set of conditional attributes as all the attributes to be reduced and set the target attribute set as an empty set. Secondly, a conditional attribute in the attribute set to be reduced is copied to the target attribute set, and the lower approximation of the fuzzy rough set is obtained according to the upper and lower approximation calculation method of the nearest neighbor based on *k*-order weighted average, so as to obtain the importance of the current target attribute set to the decision attributes, and then, the added conditional attributes need to be removed from the target attribute set. Thirdly, the selection of the next attribute in the attribute set is continued to be reduced and the corresponding operation until each attribute in the attribute set to be reduced is traversed is completed, and then, the condition attribute is selected that makes the target attribute set increase the most importance to the decision attribute to join the target attribute set and delete the attribute from the attribute set to be reduced. Finally, whether the target attribute set meets the requirements is judged. If not, the qualified attributes selected from the attribute set to be reduced to the target attribute set are added. Otherwise, the attribute selection process is terminated and the final target attribute set is obtained.

### 2.3. Description of Attribute Selection Algorithm

Previously, we have introduced the secondary reduction in conditional attributes based on the similarity and maximum similarity criteria of conditional attributes and the final reduction process and related theories of attributes in the nearest neighbor region based on k-order weighted average. To effectively combine the two, reduce the dimension of network security data, and accurately extract the situation elements, this study designs the following attribute selection algorithm.

Through the above algorithm, the redundant information between condition attributes is considered, and the redundant condition attributes are deleted under the condition of ensuring the information breadth. At the same time, the membership degree of samples belonging to the real class is ensured to be the largest. It can reduce the influence of noise samples, reduce the misclassification probability of samples, and shorten the time of calculating the upper and lower approximation of fuzzy rough sets. The algorithm also does not need to solve the core attributes of conditional attribute set in attribute reduction, which reduces the time of feature selection to a certain extent.

## 3. Design of Situation Element Extraction Model Based on Combination Classifier

Although the traditional recognition system relying on a single classifier can achieve high recognition rate in some problems, it generally needs more samples to train, which increases the time and space cost of system training. When faced with complex problems, we cannot require a single classifier recognition system to have good recognition ability for all target categories, and the recognition system is prone to overfitting. A combined classifier recognition system can make full use of the complementary classification information of different classifiers, to overcome the shortcomings of single classifier. The construction of combined classifier recognition system mainly consists of two parts, namely, the design of classifier group and the design of fusion layer. The design of these two parts has no sequence. We can design the classifier group or the fusion layer first, but the design of these two parts must be related to each other. The classification method adopted by the classifier group should match the fusion method adopted by the fusion layer, and the output of the classifier group can be used as the input of the fusion layer. Only when the two parts are designed reasonably and combined effectively, the performance of the combined classifier recognition system can be brought into full play.

### 3.1. Design of Classifier Group in the Model

The traditional single classifier recognition system generally selects a suitable classifier to train and recognize the target according to the specific problems and expert experience. Even if multiple classifiers are used, the best one is selected by comparing these classifiers, and the remaining classifiers are discarded. Combined classifier recognition system needs to select a group of classifiers from many classifiers and effectively combine these classifiers to make full use of the complementary information between different classifiers, so as to improve the performance of the recognition system.

The design of classifier group in combined classifier recognition system is relatively simple. Generally, several classifiers that meet the corresponding requirements are selected from many classifiers to construct a classifier group through some measurement indexes. For example, in reference, a method of using the genetic algorithm to select a group of classifiers is proposed. In this method, each classifier is constructed as a gene of the genetic algorithm, and then, the chromosome of the optimal gene combination is obtained through genetic evolution; thus, a subset of classifiers is selected in the classifier set. In this study, from the recognition rate, ROC curve, learning time, and other indicators, the performance of each classifier is comprehensively considered. Four classifiers are selected from 15 commonly used classifiers, and they are constructed into a classifier group. The specific selection process will be introduced in detail in the experimental part. In addition, it has been mentioned that to make the output of the classifier contain more information, the classifier with metric output form should be selected in the process of classifier group design, so the four classifiers selected in this study are classifiers with metric output form.

Using the classifier group for target recognition can make full use of the complementary information between different classifiers without demanding a certain classifier. In this way, we can not only use fewer samples to train the classifier group and prevent the classifier group from overfitting, thus effectively improving its generalization ability, but also because of the mutual restriction between different classifiers. The search space of the solution is enlarged, and the risk of getting the local optimal solution is reduced.

### 3.2. Design of Fusion Layer in the Model

In Section 2, we have introduced six fusion methods commonly used in the fusion layer of the combined classifier recognition system. These six fusion methods can achieve good results in solving simple fusion problems, but they are faced with the complex information fusion problems. The results obtained are not obvious, and the accuracy of fusion results is lower than that of single classifier in the classifier group. To make the classification results of the classifier group output more effective fusion, this study constructs a fusion method based on random vector to improve the compression factor particle population optimization BP network. Although the method is more complex than the six fusion methods, it can improve the accuracy of classification and recognition effectively.

#### 3.2.1. Improved Compression Factor PSO Algorithm Based on Random Vector

Although the traditional particle swarm optimization method can quickly get the approximate solution of the problem through iterative operation, which shows good problem optimization ability, when facing complex problems, its particles are prone to prematurity and cannot get the optimal solution of the problem, resulting in large solution error. To effectively improve the traditional PSO method, we mainly start from two aspects: (1) some advanced theories are integrated with the PSO method to study the improved PSO method. (2) Some good performance algorithms are combined with PSO to study various combinatorial optimization methods. Here are two classic improved PSO methods.

(1) PSO method with inertia weight: in order to improve the global optimization ability of the traditional PSO method, the weight with inertia was added to the particle swarm optimization method by Shi in 1998, which makes its performance better [35]. The specific form of the improved PSO method is as follows:
  (13) $$\begin{array}{c} V_{i}^{k+1}=w\cdot V_{i}^{k}+c_{1}\cdot r_{1}\cdot \left(pbest_{i}^{k}-X_{i}^{k}\right)+c_{2}\cdot r_{2}\cdot \left(gbest^{k}-X_{i}^{k}\right),\\ X_{i}^{k+1}=X_{i}^{k}+V_{i}^{k+1}, \end{array}$$
where *w* is the inertia weight. When *w*=1, this method is the traditional PSO method; when *w* is large, this method will search for the approximate solution globally to prevent premature particles, but it is easy to skip the optimal solution; and when *w* is small, the method will search for the optimal solution in the local solution space and accelerate the convergence speed, but it is easy to get the local optimal solution.
Some experts and scholars have studied the value of *w* inertia weight and put forward two common methods.
  ① The method of inertia weight decreasing linearly is as follows:
    (14) $$\begin{array}{c} w=w_{\max}-\frac{t\cdot \left(w_{\max}-w_{\min}\right)}{t_{\max}}. \end{array}$$
  Among them, *w*_max_ represents the maximum value that *w* can obtain, which is generally set as 0.9, *w*_min_ represents the minimum value that *w* can obtain, which is generally set as 0.4, *t* represents the number of current iterations of the population, and *t*_max_ represents the total number of iterations of the population.
  The above method can ensure that the value of *w* decreases gradually when the number of iterations increases. In the early stage of iteration, it can ensure to find the approximate solution globally and lock the position of the approximate solution as soon as possible, to prevent premature particles to a certain extent; in the later stage of iteration, it can ensure that the local optimal solution is searched carefully and the convergence speed is accelerated.
  ② The adaptive value method of inertia weight is as follows:
    (15) $$\begin{array}{c} w=\left\{\begin{array}{cc} w_{\min}+\left(w_{\max}-w_{\min}\right)\cdot \frac{f-f_{\min}}{f_{avg}-f_{\min}}, & f\leq f_{avg},\\ w_{\max}, & f>f_{avg}, \end{array}\right. \end{array}$$
  where *f* is the fitness of the corresponding particles, *f*_min_ and *f*_*avg*_ are the minimum and mean fitness of all particles under the current iteration number. When the fitness of particles is better than the average of all particles, it means that the particle is near the optimal solution. When *w* is small, the particle searches locally. On the contrary, it shows that it is far away from the optimal solution, and when *w* is larger, the particle carries out the global search.
  By using the fitness value of each particle to control the inertia weight of each particle, the difference between particles can be ensured, the optimal solution can be searched more comprehensively, and the premature of particles can be prevented to a certain extent.
(2) PSO algorithm with compression factor is as follows:

(16) $$\begin{array}{c} V_{i}^{k+1}=\varphi \cdot \left\{V_{i}^{k}+c_{1}\cdot r_{1}\cdot \left(pbest_{i}^{k}-X_{i}^{k}\right)+c_{2}\cdot r_{2}\cdot \left(gbest^{k}-X_{i}^{k}\right)\right\},\\ X_{i}^{k+1}=X_{i}^{k}+V_{i}^{k+1}, \end{array}$$

where *ϕ* is the compression factor:

(17) $$\begin{array}{c} \varphi =\frac{2}{\left|2-C-\sqrt{C^{2}-4C}\right|},\\ C=c_{1}+c_{2}>4. \end{array}$$

Although PSO with inertia weight can improve convergence speed and reduce the risk of getting local solution of the problem, it will lose the ability to explore the new solution space due to too small inertia weight in the later iteration period. PSO method with compression factor can effectively avoid this problem and improve the local exploration ability of the method, the better constraint particle flying to the optimal solution.

Although the performance of PSO method with compression factor is good, it can solve many optimization problems, but when it faces high-dimensional or complicated optimization problems, the solution may be local optimal. To solve this kind of complex nonlinear problem efficiently, this study introduces a compression factor PSO method based on random vector.

If the solution space of a problem is n-dimensional, the iterative optimization process can be expressed as follows:

(18) $$\begin{array}{c} V_{i}^{k+1}=\varphi \cdot \left\{V_{i}^{k}+c_{1}\cdot r_{1d}^{k}\cdot \left(pbest_{i}^{k}-X_{i}^{k}\right)+c_{2}\cdot r_{2d}^{k}\cdot \left(gbest^{k}-X_{i}^{k}\right)\right\},\\ X_{i}^{k+1}=X_{i}^{k}+V_{i}^{k+1}, \end{array}$$

where *r*_1*d*_^*k*^ and *r*_2*d*_^*k*^ represent two d-dimensional random vectors of the *k*th iteration, and each element of *r*_1*d*_^*k*^ and *r*_2*d*_^*k*^ belongs to [0,1].

This compression factor PSO method based on random vector not only has the advantage of iterative optimization of compression factor PSO method but also makes the optimization information of the previous generation of particles affect the current speed of the particles randomly through the control of random vector, to increase the differences among particles and effectively suppress the method to get the local optimal solution, further enhance the ability of particle to explore new regions, and improve the convergence speed of the method.

#### 3.2.2. Structure Description of Fusion Layer

Research has shown that if the output form of each classifier in the classifier group is metric output form, we can use neural network as the fusion method of fusion layer to realize the fusion decision. Because BP neural network has a simple structure, it is relatively easy to implement and has good performance, so this study uses it as a fusion decision method. In the optimization of BP network, the derivative of error is generally used to update the parameters in the network by back propagation. The problem solution obtained by this method of updating the parameters by gradient descent is easy to be locally optimal, so it cannot well approximate the real solution of the problem [36]. To solve this problem, this study uses the compression coefficient PSO method based on random vector to optimize the parameters of BP neural network and realizes the fast solution of parameters under the condition of reducing the computational complexity.

Because the output result of each classifier in the classifier group is the class information of the input sample, the output result of the classifier group can be regarded as the extended features of the identified sample, but such extended features are obtained through the complex transformation of the classifier and cannot fully represent the information of the sample. In order to input more information into BP fusion neural network and improve the accuracy of fusion decision, this study inputs the original features of samples and the output results of classifier group to the fusion layer, and its specific structure is shown in Figure 4. The application process of fusion layer is mainly divided into the following stages: firstly, the improved compression factor PSO method based on random vector is used to iteratively optimize the relevant parameters of BP neural network, and the trained BP fusion neural network is obtained. Then, the network security data and the corresponding results of the classifier group are input to the BP fusion network, and the BP fusion network classifies the input data to get the final fusion result. Finally, the fusion results are compared with the real value to judge the accuracy of network situation element extraction.

### 3.3. Extraction Process of Situation Elements Based on Combined Classifier

The use of the network situation element extraction system based on the combination classifier is mainly divided into two stages: training and target recognition. In the process of training, we need to train each classifier in the classifier group with network security samples; then, the optimized classifier group is used to identify the target of the network security training samples; finally, the recognition results of the classifier group and the corresponding training samples are input into BP neural network. The parameters of BP neural network are optimized using the improved compression factor PSO algorithm based on random vector, and the optimized BP fusion network is obtained. In the process of classification recognition, the first step is to input the data set of network security test into the classifier group to get the target recognition result of the classifier group to the test set; then, the target recognition results obtained by the classifier group and the corresponding network security samples are input into the fusion layer to get the final fusion recognition results; finally, the fusion recognition results are evaluated as network situation elements to verify the accuracy of extraction. The specific process is shown in Figure 5.

## 4. Experiment and Analysis

### 4.1. Experimental Environment and Data

The specific hardware environment for simulation is as follows: the CPU used is 2.60 GHz Intel Core-i5 3200M, the graphics card used is 2 GB NVIDIA GT 720M, the capacity is 12.0 GB RAM, and the capacity is 128 GB (solid state) + 500 GB (mechanical) hard disk.

The specific programming environment for simulation is as follows: Win 7 (64 bit) desktop system, PyCharm of 2019.1, Python of 3.7, TensorFlow of 1.15.1, and Keras of 2.3.1.

The experiment uses the authoritative and classic NSL-KDD data set, which is an improved version of KDD99 data set and corrects some defects of the original data set. The specific improvements of the data set are as follows: (1) the redundant samples in the original data set are deleted, which inhibits the overlearning of some samples to a certain extent and improves the accuracy of recognition. (2) The number of samples of each category is inversely proportional to the percentage of samples of different categories in the original data set, which inhibits the overlearning of some categories to a certain extent and makes different recognition technologies perform better on the data set. (3) It is reasonable to set the number of training samples and test samples and the proportion of sample categories between them, so that the recognition results of training samples and test samples are consistent and comparable. Each sample in the NSL-KDD data set contains 41 conditional features and 1 decision feature. Conditional features are composed of 7 discrete features and 34 continuous features. Although the data set cannot fully reflect the current network situation, it is still the authoritative data set used by researchers to measure the advantages and disadvantages of network situation element extraction methods.

The composition of records in NSL-KDD data set is reasonable. The total number of training samples is 25973, including 67343 normal samples and 58630 abnormal samples; the total number of samples in the test set is 22544, including 9711 normal samples and 12833 abnormal samples. This data structure solves the problem of uneven distribution of sample categories to a certain extent, which makes the recognition algorithm easier to perform, and the results are more effective. There are 21 attack modes in the training sample set, and in addition to these attacks, there are 16 new attack modes in the test sample set [37]. These attack modes can be divided into four types, and their specific distribution is shown in Table 1. The training sample set and test sample set are classified according to the attack type, and the specific classification is shown in Table 2.

### 4.2. Preparation of Experiment and Setting of Parameters

#### 4.2.1. Pretreatment of Experimental Data

① Character Data Digitization: in addition to numerical data, there are four kinds of character data (protocol_type, service, flag, label) in each sample of experimental data. To unify the standard and meet the experimental requirements, the first three of the four character data are directly converted into numerical data; for example, the value of TCP in the protocol_type condition attribute is assigned to 1, the value of UDP is assigned to 2, and the value of ICMP is assigned to 3; secondly, label data are classified according to attack types and then converted into numerical data directly; finally, the transformed label data are encoded by one hot.
② Standardization: we standardize the sample set to prevent the extreme value or outlier of the sample from affecting the experimental results.
③ Normalization: we normalize the sample set to unify the dimensions of the sample.

#### 4.2.2. The Determination of Classifiers in Classifier Group

To select several classifiers with good performance from some classifiers to construct a classifier group, 15 classical classifiers based on different principles are optimized with training samples; then, the test samples are input into 15 optimized classifiers, and the classifiers classify them, respectively; finally, four classifiers with better comprehensive performance are selected to construct a group of classifiers.

First of all, it is necessary to select the classifier with high recognition rate for U2R and R2L attack types. Because the samples of U2R and R2L attack types in the training data set are relatively small, most classifiers have the problem of under learning. If the selected classifier has a low recognition rate for both types of attacks, the fusion layer will also get a low recognition rate when fusing the recognition results, which will affect the performance of the combined classifier system; secondly, to ensure the stability of the classifier in different states, we need to choose the classifier with relatively large AUC coefficient (the area formed by ROC curve and *X* axis is relatively large); finally, considering the performance of the classifier group, it needs less training time and relatively high total recognition rate to select the classifier.

Through the above process, the classifier training and recognition in Table 3, and the ROC curve and AUC coefficient of the classifier in Figure 6, this study selects MLP classifier, k-neighbor classifier, logistic regression, and random forest classifier from 15 classical classifiers to construct the classifier group.

#### 4.2.3. Selection of Experimental Parameters

In the process of secondary reduction in conditional attributes, the initial value of clustering threshold is 0.5 and the step size is 0.01, which increases gradually until the termination condition is satisfied. In the construction process of fusion layer, the particle number of the improved compression factor PSO method based on random vector is set to 50, the values of *c*_1_ and *c*_2_ are set to 2.05, the maximum number of iterations is set to 200, and the recognition rate of samples is taken as a function of particle fitness; the activation function in the network is set to sigmoid function, the number of nodes in the output layer is set to 5, and the number of nodes in the input layer and the hidden layer depends on the specific problem.

### 4.3. Experimental Results and Analysis

We need to build the system according to the design process in Section 4. The previous construction of classifier group has been completed, so let us build the fusion layer.

To show the performance advantages of the improved compression factor PSO method based on random vector in the process of constructing fusion layer, this study compares the proposed improved PSO method with the other two PSO methods, and the results are shown in Table 4. All attributes of NSL-KDD data samples are used in the experiment, so it is necessary to input 20 extended attributes generated by classifier group and 41 conditional attributes of samples into BP fusion neural network; that is, the number of input layer nodes should be set to 61, and the number of hidden layer nodes should be set to 17 temporarily according to the experience. Let the particle number of the three methods be 50 and the maximum number of iterations be 200. *c*_1_ and *c*_2_ of the PSO method based on linear decreasing inertia weight are set to 1.4962, and *c*_1_ and *c*_2_ of the other two PSO methods are set to 2.05.

Compared with the other two PSO methods, the approximate solution obtained using the improved compression factor PSO method proposed in this study is more close to the optimal solution, which improves the recognition rate and the effect of the system. The effectiveness of the improved PSO method is verified.

The improved PSO method can optimize BP fusion neural network to achieve good results. To improve the performance of the network, we need to compare the network performance under different numbers of hidden layer nodes, so as to find the best hidden layer junction number. The experimental results show that, when the number of hidden layer nodes is 18, the sample recognition rate of the system is the highest, so the number of hidden layer nodes should be set to 18.

After constructing the target recognition system of combined classifier, to verify its effectiveness, this study designs three comparative experiments.

First, the recall rate of the target recognition system of the combined classifier is compared with that of the single classifier in the classifier group, and the results are shown in Table 5.

It can be seen that the combined classifier target recognition system is superior to the single classifier in the classifier group in both the total recognition rate and the recognition recall rate of each attack category, which proves that the combined classifier in this study is better than other single classifiers in the classifier group, thus proving the effectiveness of the combined classifier system in this study.

Second, the output of the classifier group is fused through the fusion layer designed in this study and the fusion method mentioned in Section 2. The results are shown in Table 6.

It can be seen that although the six classical fusion methods are relatively simple in calculation and the recognition rate of some categories is higher than that of the fusion method in this study, the recognition recall rate of each attack category is lower than that of the fusion method in this study, which can also be proved from the average F1 value of macro (the average F1 value of each attack category). Moreover, the total recognition rate of the six classical fusion methods is lower than that of the single classifier of the classifier group, so in the face of complex problems, the classical fusion methods not only cannot well fuse the output of the classifier group but also can play a counterproductive role. Compared with the six classical fusion methods, the fusion method proposed in this study not only greatly improves the total recognition rate but also greatly improves the F1 value of each category; that is, it ensures a higher recognition rate and recall rate at the same time, which proves that the fusion method proposed in this study is effective.

Third, to further prove the effectiveness of the combined classifier system, this study compares it with several current classic neural networks. In the experiment, the number of iterations of each recognition system is set to 200, and the results are shown in Table 7.

It can be seen from the table that the above target recognition systems have fully studied the training set, but the recognition effect of the first four neural networks on the test set is not ideal; that is, the generalization rate is not high, and the recognition rate of the test set and the recall rate of each attack category have been significantly improved by the combined classifier system in this study, which proves the feasibility of the recognition system in this study.

The value of num_outbound_cmds attribute in NSL-KDD data set is all zero, which has no effect on situation element extraction, so it should be deleted before attribute reduction. The secondary attribute set obtained by the attribute secondary reduction method in this study is shown in Table 8, and the final attribute set obtained by the attribute final reduction method in this study is shown in Table 9.

To verify the effectiveness of the proposed attribute reduction method, three comparative experiments are designed.

First, the four classifiers in the classifier group are optimized using the training samples that are not reduced and the training samples that are reduced by the feature selection method in this study. Then, the four classifiers are identified using the test samples that are not reduced and the test samples that are reduced by the method in this study.

It can be seen from the corresponding experimental results in Table 10 that the training time of the classifier is reduced by attribute reduction, and the recognition rate of three of the four classifiers has been improved to varying degrees, which proves that the attribute reduction method proposed in this study is feasible.

Secondly, the feature selection methods in this study are compared with those of literature [38] and document [39], and the results are shown in Table 11.

It can be seen that the performance of training and recognition using the data set reduced by the method of this study is better than the other two methods. It shows that the attribute reduction method is effective.

Thirdly, the combination classifier system is trained and recognized with the original data set and the data set is reduced by the attribute reduction method to improve the performance of the attribute reduction method. Because the feature of the sample becomes 12 after feature reduction, the node number of the input layer of BP network should be adjusted to 32, and the optimal node number of the hidden layer needs to be determined again. The experimental results show that the optimal node number is 13.

After the combined classifier system used before and after attribute reduction is constructed, the corresponding sample sets are used to train and identify them, respectively. The corresponding experimental results are given in Table 12.

It can be seen that although attribute reduction can reduce the recall rate of DoS attack recognition, it can be ignored. Therefore, using the attribute reduction method in this study can further improve the performance of the combination classifier system and extract more accurate situation elements, which proves the effectiveness of the attribute reduction method in this study and also proves that it is feasible to extract situation elements combined with the combination classifier.

## 5. Conclusion

The main contributions of this study are as follows:

1. The relevant theories of situation element extraction are summarized. The classical situation element extraction process is analyzed and improved, the corresponding algorithm is designed, and a situation element extraction framework based on fuzzy rough set and combined classifier is constructed.
2. To delete redundant information between conditional attributes on the premise of ensuring information breadth and data classification ability, an attribute secondary reduction method based on conditional attribute similarity and maximum similarity criterion is proposed. Firstly, the similarity matrix of conditional attributes is obtained by this method, and then, the conditional attributes are clustered using the direct clustering method and reasonable threshold. Finally, the representative attributes are selected using the maximum similarity criterion to complete the secondary reduction in conditional attributes.
3. To ensure the maximum membership of the samples belonging to the real category, reduce the probability of misclassification, and reduce the influence of noise samples, an upper and lower approximation calculation method of the nearest neighbor domain based on *k*-order weighted average is proposed and applied to the fuzzy rough set theory. A heuristic reduction method for the secondary conditional attributes is designed to obtain the final reduced attribute set.
4. To establish a better combined classifier, this study selects 4 classifiers with good personality from 15 classical classifiers to construct a classifier group according to some measurement indexes of the classifier. Then, the improved PSO method is used to optimize the BP neural network as the fusion layer of the combined classifier, so as to complete the construction of the model.
5. The attribute selection method and combined classifier model in this study are coded, and a variety of comparative experiments of fusion method, attribute selection method, and target recognition system are carried out on the authoritative NSL-KDD data set to verify the effectiveness and feasibility of the network situation element extraction model based on fuzzy rough set and combined classifier.

At the same time, this study also has some shortcomings:

1. The model is applied to a more real network environment, so as to further test the advantages and disadvantages of the situation element extraction method.
2. In the process of attribute reduction, although some complex computation is avoided, it still needs a certain amount of computation. In the future research, we should further explore measures to improve the efficiency of attribute selection methods or make effective attempts on parallel attribute reduction.
3. In the process of building classifier group, we explore more reasonable construction methods, to make the selected classifier group better and further improve its performance.
4. The extracted network situation elements are effectively applied to situation understanding and prediction to realize its real value.

## Figures and Tables

**Figure 1:** Secondary cycle reduction process of conditional attributes.

**Figure 2:** Sample distribution diagram.

**Figure 3:** Final attribute reduction process based on improved fuzzy rough set.

**Figure 4:** Structure of fusion layer.

**Figure 5:** Extraction process of network situation elements based on combined classifier.

**Figure 6:** ROC curve and AUC coefficient of classifier.

**Algorithm 1:** Based on conditional attribute similarity and improved fuzzy rough set attribute selection algorithm.

**Table 1:** Specific classification of attack modes.

Attack type	Attack mode
DOS	apache2, back, land, mailbomb, Neptune, pod, processtable, smurf, teardrop, udpstor
Probe	ipsweep, mscan, nmap, portsweep, saint, Satan
R2L	ftp_write, guess_password, imap, multihop, named, phf, sendmai, snmpgetattack, snmpguess, 、warezmaster, worm, xlock, xsnoop
U2R	buffer_overflow, httptunnel, loadmodule, perl, ps, rootkit, sqlattack, xterm

**Table 2:** Sample distribution of data set.

Data set	Normal	DOS	Probe	R2L	U2R
Training set	67343	45927	11656	995	52
Test set	9711	7458	2421	2754	200

**Table 3:** Comparison of training and recognition of classifiers.

Classifier	Total recognition rate	Normal recall	Probe recall	DOS recall	U2R recall	R2L recall	Train time (s)
Linear SVC	0.7574	0.6575	0.8469	0.9637	0.8889	0.4444	13.12
SVC	0.7468	0.6541	0.7965	0.9544	0.8333	0.3846	105.23
Complement NB	0.6288	0.6372	0.3795	0.8400	0.0000	0.0000	0.06
MLP	0.7505	0.6534	0.7916	0.9648	0.7222	0.9404	191.03
K-Neighbors	0.7548	0.6602	0.8108	0.9573	0.8462	0.9322	43.62
Logistic regression	0.7588	0.6528	0.8914	0.9690	0.7500	0.5000	54.68
SGD (log)	0.7423	0.6384	0.8776	0.9665	0.0000	0.4444	2.71
SGD (modified_huber)	0.7549	0.6552	0.8466	0.9628	0.6667	0.2222	3.01
Decision tree	0.7724	0.6874	0.8569	0.9209	0.3125	0.7736	2.53
Extra tree	0.7309	0.6540	0.7639	0.9471	0.5385	0.4471	0.30
Gradient boosting	0.7241	0.6357	0.7112	0.9582	0.9167	0.1321	290.57
AdaBoost	0.7241	0.6781	0.5629	0.8576	0.2500	0.8202	15.54
Random forest	0.7527	0.6478	0.8783	0.9643	1.0000	0.9623	23.73
Bagging	0.7429	0.6560	0.7729	0.9216	0.4000	0.8304	18.11
Extra trees	0.7425	0.6429	0.8372	0.9587	0.0000	0.8333	23.65

**Table 4:** Comparison of three PSO methods.

PSO method	System recognition rate	Mean square error of the system
PSO method based on linear decreasing inertia weight	0.8769	0.042
Classical compression factor PSO method	0.9007	0.028
Improved compression factor PSO method based on random vector	0.9302	0.018

**Table 5:** Comparison of recall rate between combined classifier and single classifier in classifier group.

Classifier	Total recognition rate	Normal recall	Probe recall	DOS recall	U2R recall	R2L recall
MLP	0.7505	0.9722	0.6072	0.7763	0.0650	0.0744
K-Neighbors	0.7548	0.9777	0.6584	0.7788	0.0550	0.0399
Logistic regression	0.7588	0.9725	0.7361	0.7869	0.0150	0.0033
Random forest	0.7527	0.9751	0.6109	0.8002	0.0050	0.0185
Combined classifier	0.9449	0.9876	0.9996	0.9983	0.2900	0.6304

**Table 6:** Comparison of results between fusion methods.

Fusion method	Total recognition rate	Normal recall	Probe recall	DOS recall	U2R recall	R2L recall	Macro-average F1 value
Voting method	0.7343	0.6318	0.8534	0.9641	0.6667	0.8125	0.4687
Maximum rule	0.7417	0.6449	0.8034	0.9615	0.8462	0.9496	0.4984
Minimum rule	0.7424	0.6454	0.8053	0.9623	0.8462	0.9640	0.4993
Mean method	0.7482	0.6466	0.8491	0.9637	0.8333	0.9528	0.4990
Median method	0.7530	0.6513	0.8479	0.9645	0.8000	0.9697	0.4986
Product rule	0.7425	0.6457	0.8060	0.9618	0.8000	0.9524	0.4933
Improved fusion method	0.9449	0.9670	0.7608	0.9925	1.0000	0.8962	0.8053

**Table 7:** Comparison of recognition recall rate between combined classifier and neural network.

Target recognition system	Total recognition rate	Normal recall	Probe recall	DOS recall	U2R recall	R2L recall	Training loss
CNN	0.7373	0.9701	0.5184	0.7741	0.0150	0.0641	0.0155
DNN	0.7648	0.9761	0.5973	0.8284	0.0150	0.0494	0.0120
GRU	0.7417	0.9719	0.5820	0.7659	0.0450	0.0559	0.0082
LSTM	0.7523	0.9631	0.6332	0.7891	0.0450	0.0654	0.0079
Combined classifier system	0.9449	0.9876	0.9996	0.9983	0.2900	0.6304	0.0054

**Table 8:** Attribute secondary reduction set.

Method	Number of attributes after reduction	Attribute collection
Attribute secondary reduction	26	Duration, service, flag, src_bytes, dst_bytes, land, wrong_fragment, hot, num_compromised, root_shell, su_attempted, num_shells, num_access_files, is_guest_login, count, srv_count, serror_rate, srv_rerror_rate, same_srv_rate, diff_srv_rate, srv_diff_host_rate, dst_host_count, dst_host_same_srv_rate, dst_host_diff_srv_rate, dst_host_same_src_port_rate, dst_host_rerror_rate

**Table 9:** Final attribute reduction set.

Method	Number of attributes after reduction	Attribute collection
Attribute final reduction	12	Service, flag, root_shell, count, srv_count, serror_rate, srv_rerror_rate, same_srv_rate, diff_srv_rate, dst_host_count, dst_host_same_src_port_rate, dst_host_rerror_rate

**Table 10:** Comparison of recognition performance before and after feature selection.

Classifier	Before feature selection		After feature selection	
	Total recognition rate	Training time (s)	Total recognition rate	Training time (s)
MLP	0.7505	191.03	0.7991	106.42
K-Neighbors	0.7548	43.62	0.7649	30.44
Logistic regression	0.7588	54.68	0.7107	38.65
Random forest	0.7527	23.73	0.7624	10.60

**Table 11:** Comparison of experimental results of different attribute reduction algorithms.

Attribute reduction method	Number of attributes after reduction	Total recognition rate			
		MLP	KN	LR	RF
Method of reference [38]	10	0.7077	0.7102	0.6702	0.7214
Method of reference [39]	16	0.7514	0.7512	0.7074	0.7053
The method of this study	12	0.7991	0.7649	0.7107	0.7624

**Table 12:** Performance of combined classifier system before and after attribute reduction.

Combined classifier system	Total recognition rate	Normal recall rate	Probe recall rate	DOS recall rate	U2R recall rate	R2L recall rate	Training loss
Before attribute reduction	0.9449	0.9876	0.9996	0.9983	0.2900	0.6304	0.0054
After attribute reduction	0.9623	1.0000	1.0000	0.9981	0.5450	0.7633	0.0032

## Data Availability

The data sets used and analyzed during this study are available from the corresponding author on reasonable request.
